The article "Inhibitory Effects of Rhein on Renal Interstitial Fibrosis via the SHH-Gli1 Signal Pathway" was published in 2022. Journal: Evid Based Complement Alternat Med.

# Inhibitory Effects of Rhein on Renal Interstitial Fibrosis via the SHH-Gli1 Signal Pathway

**DOI:** 10.1155/2022/4398265

**Published:** 2022-08-05

**Authors:** Yan Luo, Juan Jiang, Junxiong Cheng, Chen Xuan, Yu Xiong, Weijian Xiong, Wenfu Cao, Ying Li

**Affiliations:** ^1^Chongqing Traditional Chinese Medicine Hospital, Chongqing 400021, China; ^2^Chongqing Key Laboratory of Traditional Chinese Medicine for Prevention and Cure of Metabolic Diseases, Chongqing 400016, China; ^3^College of Traditional Chinese Medicine, Chongqing Medical University, Chongqing 400016, China; ^4^Chongqing University Cancer Hospital, Chongqing, China

## Abstract

**Background:**

Rhein is the main extract of *Rheum palmatum* L., which has been proved to improve the renal function of chronic kidney disease, but its mechanism is not clear. Therefore, this experiment explored the potential pharmacological effect of rhein on renal interstitial fibrosis rats.

**Methods:**

This study explores the potential pharmacological action of rhein. In this work, we investigate the potential pharmacological action of rhein in unilateral urethral obstruction (UUO) rats. Thirty Sprague Dawley rats were randomly divided into three groups: sham, UUO, and rhein (rhein-treated UUO rats) groups. The left ureters of the UUO group rats were exposed and bluntly dissected. The rhein group rats were administered an intragastric gavage of rhein (2 mg·kg^−1^·d^−1^) for 14 d. Kidney function-related indicators were monitored in these rats, while indexes of pathologic aspects were determined histologically. The expression of *α*-SMA, TGF-*β*1, SHH, Gli1, and Snail was quantified using real-time polymerase chain reaction and western blotting. The NRK-49F cells were incubated with and without SHH (100 ng·ml^−1^) for 48 hours. The SHH-activated NRK-49F cells were incubated with cyclopamine (CNP, 20 umol L^−1^) or rhein (1 ng·ml^−1^). The Gli1 and Snail mRNA and protein level were detected.

**Results:**

In the in vivo experiment, the results exhibited that UUO caused renal pathological damages. However, these changes could be significantly reversed by the administration of rhein. Compared with the untreated UUO group, the rhein group showed reduced kidney tubular atrophy and necrosis, interstitial fibrosis, hyperplasia, and abnormal deposition of extracellular matrix. Rhein reduced the RNA and protein expression of SHH, Gli1, and Snail of the UUO rats. In the in vitro experiment, CNP or rhein treatment decreased the expression of Gli1 and Snail on mRNA and protein levels in SHH-induced NRK-49F cells, suggesting that CNP or rhein suppresses SHH-induced NRK-49F activation. Taken together, these results demonstrated that rhein suppresses SHH-Gli1-Snail signal pathway activation, with potential implications for the treatment of renal fibrosis.

**Conclusions:**

Treatment with rhein remarkably ameliorated renal interstitial fibrosis in UUO rats by regulating the SHH-Gli1-Snail signal pathway.

## 1. Introduction

Currently, chronic kidney disease (CKD) is the 16^th^ cause of death worldwide. It has become a prominent public health issue in the world, with a global incidence of approximately 10–15% [1]. Once developed in irreversible end-stage kidney disease (ESRD), they can only be treated with dialysis and kidney transplants. Kidney fibrosis is the buildup of scar within the parenchyma, and it represents the common final pathway of nearly all chronic and progressive nephropathies [2]. It has been proved that transforming growth factor *β*1 (TGF-*β*1) secreted by renal tubular cells. TGF-*β*1 was identified to be the grandmaster that elicits numerous signals, which culminate in fibrosis and renal parenchymal loss. Importantly, TGF-*β*1 can induce activated renal interstitial fibroblasts, myofibroblasts, which are characterized by *α*-smooth muscle actin (*α*-SMA) expression [3]. The increased expression of TGF-*β*1 and *α*-SMA is a manifestation of epithelial-to-mesenchymal transition (EMT). In the formation of renal interstitial fibrosis (RIF), EMT is believed to play an important role in organ fibrosis [4], chronic inflammation [5], tissue reconstruction [6], and various fibrotic diseases [7].

In recent years, SHH signal pathway has been proved to be closely related to tissue fibrosis, which involves liver, bile, lung, kidney, and other organs. It was found that SHH was almost not expressed in normal adult kidneys, while the expression of SHH in renal tubular epithelial cells was significantly upregulated in patients with CKD caused by various causes. This result has also been confirmed in various rat renal fibrosis models such as unilateral ureteral obstruction (UUO) [8]. These results suggest that SHH signal pathway activation is a common pathological result of various renal diseases. Consequently, inhibition of myofibroblast activation and SHH signal pathway may be an effective strategy to prevent renal fibrosis.

*Rheum palmatum* L., a type of traditional Chinese herb defecation-promoting purgative medicinal, has bitter and cold medicinal properties [9]. Rhein is a main bioactive component of *Rheum palmatum* L., which has been widely used for the treatment of chronic kidney-related diseases in the clinic [10]. Recent studies have shown that rhein has potent anti-autophagy [11], anti-apoptosis [12], and antifibrosis [13]. Rhein can remarkably improve renal interstitial fibrosis in vivo whether its potential mechanism may be related to the inhibition of SHH-Gli1-Snail signal pathway.

To investigate the mechanism of rhein and understand its potential antifibrosis effect on renal, the UUO model was used to simulate renal interstitial fibrosis in rats. Here, UUO causes subacute renal injury characterized by tubular cell injury, interstitial inflammation, and fibrosis, a well-known model to induce renal fibrosis in vivo [14]. The in vivo study aimed to investigate the pathological changes of renal fibrosis, and the effects of rhein on the expression of SHH, Gli1, and Snail proteins were analyzed. And the in vitro study aimed to investigate rhein on the expression of Gli1 and Snail on mRNA and protein levels, which activated with human SHH protein and rat NRK-49F cells. The activated renal fibrosis by SHH signal pathway and the protective mechanism antifibrosis of rhein were discussed in this study.

## 2. Materials and Methods

### 2.1. Animals and Cells

Seven-week-old thirty clean-grade male SD rats (200 ± 20) g were approved by the Animal Experimental Ethics Committee of Chongqing Medical University (Chongqing, China; Animal license No. SCXK:2018–0003) and performed by the Guidelines of the Animal Care Committee of Chongqing Medical University. Normal rat kidney interstitial fibroblasts (NRK-49F) were purchased from the American Type Culture Collection (ATCC, Manassas, VA).

### 2.2. Reagents and Instruments

Reagents and instruments used for this study are as follows: rhein (Rhawn, Shanghai, China); cyclopamine (Selleck Chemicals, Houston, USA); human SHH protein (StemRD Inc, USA); antibodies against TGF-*β*1 and *α*-SMA (Servicebio, Wuhan, China); antibodies against SHH, Gli1, Snail, and GAPDH (Affinity Biosciences, Jiangsu, China); PVDF membrane, BCA Protein Assay Kit, BeyoECL Moon kit (Beyotime Biotechnology, Shanghai, China); TRIzol (Takara Bio, Shiga, Japan); primers for qPCR (Servicebio, Wuhan, China); AU400 automatic biochemical analyzer (OLYMPUS, Tokyo, Japan); BX51T-PHD-J11 microscope (OLYMPUS Company, Tokyo, Japan); image acquisition system CMOS (OLYMPUS Company, Tokyo, Japan); Image-Pro Plus (National Institutes of Health, Bethesda, USA); and TEM (JEM1400PLUS, JEOL, Tokyo, Japan).

### 2.3. Animal Experiments

After one week of adaptive breeding, thirty male SD rats were randomly divided into three groups: sham group (sham operation rats), UUO group, and rhein group (rhein-treated UUO rats) with 10 rats in each group. Besides the sham group, the other two groups underwent the same surgical procedures to establish UUO model rats: after anesthesia with 2% sodium pentobarbital, the kidneys of rats were exposed, and then, the left ureter was double-ligated. Rats in the sham group were performed with sham operations without being ligated on left ureter. The rhein group rats were administered at 2 mg·kg^−1^·d^−1^, and rhein was dissolved in 0.5% carboxymethyl cellulose sodium (CMC-Na+) in H_2_O, through intragastric gavage for 14 d. The rats in the sham and model groups received intragastric administration of 0.5% CMC-Na+ (2 mg·kg^−1^·d^−1^) for 14 d. After 2 weeks, all rats were sacrificed. Blood and tissues were harvested from rats that were fasted for 12 h.

### 2.4. In Vitro Experiments

The NRK-49F cells were treated with 10% fetal bovine serum, 100 U/mL penicillin, 100 mg/L streptomycin, and 37°C in 5% CO_2_ in the DMEM medium. Rhein was dissolved by dimethyl sulfoxide (DMSO). The cells were divided into four groups: the control group without any treatment, the SHH group (100 ng/L human SHH protein), the SHH + Rhein group (100 ng/L human SHH protein + 1 ng/ml rhein), and the SHH + CPN group (100 ng/L human SHH protein + 20 umol/L cyclopamine). When the cells grew to 80% ∼ 90% fusion, the activation of cells was induced for 48 hours by 100 ng/L human SHH protein. The culture medium was discarded, the corresponding serum and reagents were added in each group, and the cells were collected 24 hours later. The expression of Gli1 and Snail in vitro was evaluated by western blot analysis or RT-PCR.

### 2.5. Histopathological Analysis of Renal Tissue

Rat renal tissue was first fixed in 4% paraformaldehyde for 48 h, embedded in paraffin, and further sectioned. The 3-*μ*m-thick sections obtained were dewaxed, treated with gradient ethanol, and stained with hematoxylin-eosin (HE), Masson, and periodic acid-Schiff (PAS) stains. Pathological analysis of glomeruli and tubules was performed using a light microscope.

The interstitial score of the renal tubules was analyzed at a 200× magnification; ten tubules per visual field were observed. According to the range of renal tubular atrophy, tubular type, stromal cell infiltration, and fibrosis, scores from 0 to 3 were assigned: 0 for none; 1 for less than 25%; 2 for 25–50%; and 3 for 50–75% [15]. Photo images from each cortex were screened, and scores were added based on tubulointerstitial injury: tubular atrophy, tubular necrosis, and interstitial fibrosis [16, 17].

### 2.6. Electron Microscopy

The morphological and microstructural structures of kidneys, such as the glomerular basement membrane, mesangial cells, podocytes, endothelial cells, and collagen fibers in the interstitial tissue, were examined using transmission electron microscopy (TEM). The renal tissues from the rats were fixed in 2.5% glutaraldehyde and embedded in paraffin. The 70-nm-thick tissue sections were stained and observed by TEM.

### 2.7. Immunohistochemistry

The 3-*μ*m-thick renal tissue sections were incubated with citrate antigen retrieval solution for 20 min at 95°C. Thereafter, the sections were stained with a monoclonal antibody against transforming growth factor *β* (TGF-*β*1; dilution 1 : 500) and *α*-smooth muscle actin (*α*-SMA; dilution 1 : 500). The sections were incubated with goat anti-rabbit antibodies overnight and further, with a secondary antibody for 50 min. The positive areas were visualized using the DAB Kit. The integrated optical density of protein expression was calculated using the ImageJ software.

### 2.8. Real-Time PCR

According to the manufacturers' protocols, total RNA was extracted from renal tissue using TRIzol reagent, according to the manufacturer's instructions. Furthermore, RNA was reverse-transcribed into cDNA. The PCR cycling conditions were as follows: 94°C for 5 min, followed by 95°C for 30 s and 57°C for 30 s, and then 32 cycles of 72°C for 10 min. Gene expression levels were calculated from the standard curve using the expression of the glyceraldehyde 3-phosphate dehydrogenase (GAPDH) gene as a reference.

### 2.9. Western Blotting

Renal tissue proteins were extracted, quantified, and visualized by western blotting through electrophoresis, membrane transfer, and antibody incubation. Primary antibodies (1 : 1,000 dilution) against SHH, Gli1, and Snail were used, and the membranes were incubated overnight at 4°C on a shaking bed. Furthermore, the secondary antibody (1 : 2,000 dilution) was added and incubated at 37°C for 120 min. After applying the ECL color reagent and performing dark chamber exposure imaging, the gray value of the images was analyzed using ImageJ software (National Institutes of Health, Bethesda, MD).

### 2.10. Statistical Analysis

Data analysis was carried out using SPSS 17.0 software (SPSS Inc., Chicago, United States). Data are presented as mean ± standard deviation. Variables in each group were tested to determine whether they were normally distributed. The statistical analyses were performed by one-way analysis of variance followed by a least significant difference test or Dunnett's multiple comparison test. *p* < 0.05 was considered statistically significant.

## 3. Results

### 3.1. Effects of Rhein Improves Histopathological Changes

Renal fibrosis is characterized by glomerulosclerosis, renal tubulointerstitial fibrosis, renal vascular fiber sclerosis, and excessive accumulation and deposition of extracellular matrix (ECM). The pathological manifestations were renal tubular dilatation with atrophy (green arrow); renal tubular epithelial cell edema (blue arrow); cytoplasmic loose staining, lymphocyte proliferation, and infiltration (yellow arrow); endothelial cell proliferation, ECM component proliferation, renal interstitial matrix proliferation, and mesangial area expansion (orange arrow); thickening of the basement membrane (red arrow); and foot process fusion loss (brown arrow). In this research, we evaluated the pathological changes of the kidney from different perspectives by renal appearance, HE or PAS staining, and transmission electron microscopy. The positive parts of the lesions are marked with arrows in the UUO group and the rhein group. Compared with the UUO group, rhein ameliorates these pathological injuries (Figure 1).

### 3.2. The Effect of Rhein in Alleviate Renal Fibrosis

Renal fibroplasia was evaluated by Masson staining. The main components of the ECM examined the expression of TGF-*β*1 and *α*-SMA by immunohistochemistry. In Masson staining, collagen fibers are shown in blue (purple arrow). Compared with the sham group, there was a significant accumulation of collagen fibers in the kidney tissue of the UUO group. Compared with the sham group, the ECM of TGF-*β*1 and *α*-SMA expression shown in yellow was significant accumulation. These results confirm that our experimental model was successful and indicates that rhein delivery alleviates the pathological changes and renal fibroplasia observed in UUO rats (Figure 2).

### 3.3. The Effects of Rhein on SHH-Gli1-Snail Signal Pathway

The SHH signal pathway is an important pathway regulating fibrosis. Inhibition of the SHH signal pathway is associated with the inhibition of renal fibrosis. We examined the expression of SHH, Gli1, and Snail downstream in the renal. In comparison with the sham group, the expression of SHH, Gli1, and Snail of the UUO group was increased significantly (*p* < 0.01). In comparison with the UUO group, the expression of SHH, Gli1, and Snail of the rhein group was decreased significantly (*p* < 0.05). The result suggests that rhein can inhibit activation of the SHH signal pathway (Figure 3).

### 3.4. The Effects of Rhein on SHH Pathway In Vitro Experimental Results

Compared with the sham group, the expression of Gli1 and Snail in NRK-49F cells stimulated by SHH (100 ng/ml) was significantly increased. SHH markedly induced de novo Gli1 and Snail expression in renal interstitial fibroblast NRK-49F cells. The results showed that simultaneous incubation with cyclopamine (CNP, 20 umol/L) repressed SHH-initiated Gli1 and Snail expression of NRK-49F cells (*p* < 0.05). And incubation with rhein (1 ng/ml) also had the same effect as CNP (*p* < 0.05). (Figure 4).

## 4. Discussion

Rhein is one of the anthraquinone active components in *Rheum palmatum* L. *Rheum palmatum* L. is widely used in TCM as an indispensable and specific treatment for curing CKD stages 1–5 and shows good curative effects. Rhein possesses multiple pharmacological activities, including antioxidation, anticancer, antiviral, anti-inflammatory, antifibrosis, anti-hyperuricemic, and purgative effects [18, 19]. Rhein could attenuate kidney damage in diabetic rats by improving glucose metabolism abnormality, reversing insulin resistance and dyslipidemia, and effectively preventing diabetic nephropathy [20]. Numerous research suggests that rhein protected kidney through various signal pathways involvement [11, 21, 22].

Renal fibrosis is a common pathological pathway leading to end-stage renal disease. UUO surgery can cause renal pathological changes, involving periglomerular fibrosis, rupture of glomerular capillary wall in renal capsule, blood flowing into renal capsule and coagulation, resulting in proliferation of epithelial cells, proliferation of podocytes, infiltration of monocytes, production of a variety of fibrogenic cytokines, proliferation and fibrosis of fibroblasts, and inward compression of capillaries, or the fusion of glomerular capillaries and renal capsule basement membrane is called balloon adhesion, which pulls the capillaries to the renal capsule basement membrane to form glomerulosclerosis. The basement membrane of renal vesicles was thickened, renal vesicles were dilated, and capillary loops were squeezed [23]. During glomerular ischemia, the early manifestation is ischemic shrinkage, and in the late stage, due to ischemia, the capillary wall is hypoxic, resulting in increased permeability, plasma protein leakage and condensation in the renal capsule, and finally hardening. The blood supply of renal tubules comes from glomerulus, so renal tubules are more vulnerable to ischemic injury, cytoplasmic turbidity and swelling, renal interstitial edema, inflammatory cell infiltration, and renal interstitial fibrosis (RIF) [14].

Renal interstitial fibrosis (RIF) is the main pathological change of multiple chronic kidney disease (CKD). It is a common pathway that ultimately leads to end-stage renal disease (ESRD) [2, 24]. The extent and severity of RIF are highly correlated with the degree of renal dysfunction [25]. Therefore, improving RIF is of great significance to slow down and reverse the progression of CKD. The occurrence and development process of RIF mainly includes the following four links: regulation of cytokine expression, inflammatory cell infiltration, cell proliferation and epithelial-mesenchymal transition (EMT), and abnormal accumulation of extracellular matrix (ECM) [26]. EMT is a critical process of kidney fibrosis by which epithelial cells lose their epithelial characteristics and acquire the mesenchymal features, and the transformation of renal tubule epithelial cells, fibroblasts and other cells into myofibroblasts, and the formation of ECM. In the formation of RIF, EMT is believed to play an important role in organ fibrosis [4]. Renal EMT consists of four key steps: loss of adhesion between epithelial cells; newly synthesized *α*-smooth muscle actin (*α*-SMA) expression and actin recombination; rupture of basement membrane of renal tubules; and the ability of cells to migrate and invade. *α*-SMA is a specific marker of interstitial cells, which is expressed at a low level in normal tissues and organs but upregulated in tissues or cells during interstitial transdifferentiation. Studies have shown that the level of *α*-SMA-positive expression is positively correlated with the degree of tissue fibrosis, and a large amount of *α*-SMA expression is a marker of epithelial and mesenchymal cell transformation [27].

EMT in renal tubule has been demonstrated in various animal models of renal interstitial fibrosis, such as unilateral ureteral obstructive (UUO), nephropathy, and diabetic nephropathy [28]. Transforming growth factor *β*1 (TGF-*β*1) is a key player in the development of fibrosis. TGF-*β*1 is expressed in all mammalian cells and is an important cytokine to induce EMT [29]. TGF-*β* is a secretory stimulating protein, which can affect autocrine and paracrine of cells. In some cultured epithelial cells, EMT can be induced by TGF-*β*1 stimulation alone. TGF-*β* mainly includes three types, namely, TGF-*β*1, TGF-*β*2, and TGF-*β*3. TGF-*β*1 plays an important regulatory role in the occurrence and development of pathological processes, including tumor and fibrosis [30]. The present study demonstrated the fibrotic tissue and extracellular matrix were significantly increased in the UUO group. After administration of rhein, the expression of renal fibrin TGF-*β*1 and *α*-SMA decreased significantly, and the thickening of basement membrane was suppressed than that in the model group.

Activation of SHH signal pathway can induce the transformation of rat renal fibroblasts into myofibroblast phenotype. Studies have shown that sonic hedgehog (Shh) signal pathway is closely related to various organ fibroses [31]. The pathway is composed of patched SHH ligands, cell membrane receptors (Ptc), smoothened (SMO) protein, and Gli1 (Gli1, Gli2 and Gli3) downstream transcription factors. SHH can hardly be detected in normal people. When fibrosis occurs, the expression of SHH is increased, which can bind to Ptc and remove the inhibitory effect of Pct on SMO. Increased SMO expression stimulates increased downstream Gli1 expression, which enters the nucleus in full-length form and initiates transcription of target genes. Gli1 is a transcription target of hedgehog signal transduction pathway, and its activation is a reliable indicator of SHH signal activity. The SHH-Gli1 pathway participates in the process of RIF by promoting cell proliferation [32]. Studies in Gli1 knockout rats have shown that the SHH-Gli1 pathway is essential in organ fibrosis [33]. Recent studies have found that the SHH-Gli1 pathway can induce the expression of the transcription factor Snail [34], thereby activating intracellular signal transduction pathways that upregulate selected zinc finger (e.g., Snail) transcription factors and induce EMT. Studies have confirmed that Snail is an important signal molecule that triggers EMT and directly participates in the occurrence and development of RIF [32]. Study showed that TGF-*β* activated crosstalk among divergent signal pathways to Gli1 that initializes and maintains Snail expression. And Snail functions as a critical integrator of information from TGF-*β*1 signal distributed through upstream pathways [35]. TGF-*β*1 promotes the process of EMT by inducing the expression of Snail, thus promoting renal fibrosis. In the process of EMT, multiple signal pathways play a role, upregulating transcription factors and promoting mesenchymal transformation of epithelial cells. Among them, the nuclear transcription factor Snail participates in the signal transduction process of multiple signal pathways including TGF-*β*1 pathway and can induce EMT in epithelial cells, which plays an important role in the activation process of myofibroblast [36]. Lovisa [37] found that in the mouse renal fibrosis model, Snail expression was abundant in renal tubular epithelial cells within the fibrosis lesion. After the deletion of Snail gene in renal tubular epithelial cells, EMT of renal tubular epithelial cells was inhibited and renal fibrosis was alleviated (Figure 5).

The Snail family is a zinc finger transcription factor, which was first discovered in Drosophila gene in 1984. There are more than 50 members of the family. The vertebrate Snail family consists of two members: Snail (Snail1) and Slug (Snail2). Recently, it has been found that in addition to preventing expression of mesectodermal and ectodermal genes in the mesoderm anlage, Snail also take party in cellular metabolism functions, just as regulating cell differentiation, motility and apoptosis. Studies have shown that Snail can promote EMT. Snail can upregulate the expression of marker proteins *α*-SMA, myofilin, and fibronectin in mesenchymal cells. A large number of studies have confirmed that Snail is an important signal molecule that triggers EMT and directly participates in the occurrence and development of RIF. In the in vivo study, the expression of SHH, Gli1, and Snail was significantly increased in the UUO group, and the expression of SHH, Gli1, and Snail mRNA or protein was decreased after rhein treatment. The results suggest that rhein can reduce the expression of Gli1 and Snail by inhibiting SHH signal pathway, thus reducing the EMT and fibrosis in renal. The in vitro experiment showed that the activation of SHH signal pathway could significantly induce the expression of Gli1 and Snail in NRK-49F (*p* < 0.05). Adding CPN to block the SHH pathway could inhibit the upregulation of Gli1 and Snail in rat renal fibroblasts induced by SHH protein. The addition of rhein also inhibited the upregulation of Gli1 and Snail. Therefore, we hypothesized that the SHH signal pathway may promote the phenotypic transformation of NRK-49F by inducing upregulation of Gli1 and Snail expression. The antifibrosis effect of rhein may be related to the inhibition of SHH-Gli1-Snail signal pathway.

## 5. Conclusion

Our experimental data demonstrated that ingestion of rhein can modulate the pathological changes observed in UUO rats. Rhein was found to inhibit the SHH-Gli1-Snail signal pathway, which alleviated renal fibrosis in rhein-treated UUO rats. Hence, our findings reveal potential therapeutic targets for RIF and provide new perspectives on the pharmacological action of rhein during RIF treatment.

## Figures and Tables

**Figure 1:** Rhein attenuated renal histological damage. Pathological changes in the renal tissues were analyzed using renal appearance, hematoxylin-eosin (HE, ×200), periodic acid-Schiff (PAS, ×200) staining, and transmission electron microscopy (TEM, ×10,000). The pathological manifestations of renal fibrosis include renal tubular dilatation with atrophy (green arrow), renal tubular epithelial cell edema (blue arrow), lymphocyte proliferation and infiltration (yellow arrow), mesangial area expansion (orange arrow), thickening of the basement membrane (red arrow), and loss of foot process fusion (brown arrow).

**Figure 2:** Rhein improves renal fibrosis. Collagen fiber deposition (purple arrow) was observed in Masson staining. (b) ImageJ software was used to calculate the degree of renal fibrosis. ((c), (d)) Image-pro plus software was used to statistically analyze immunohistochemical staining results of TGF-*β*1 and *α*-SMA, respectively. ^*∗*^*p* < 0.05, ^*∗∗*^*p* < 0.01.

**Figure 3:** Inhibitory effect of rhein on SHH signaling pathway in UUO rats. Rhein group rats were administered rhein 2 mg·kg^−1^·d^−1^ by oral gavage for 14-d sham group, and UUO group rats were administered equal volumes of water. SHH, Gli1, and Snail protein and mRNA expression levels were determined by western blotting and RT-PCR. Data are presented as mean ± SEM. ^*∗*^*p* < 0.05, ^*∗∗*^*p* < 0.01.

**Figure 4:** Rhein inhibits SHH signaling pathway in NRK-49F cells activated by SHH. Western blot and qPCR analysis show the expression of Gli1 and Snail increased in NRK-49F cells induced by SHH (100 ng·ml^−1^) for 48 hours. The NRK-49F cells were incubated with SHH in the presence of rhein (1 ng·ml^−1^) or CNP (1 ng·ml^−1^), and the expression of Gli1 and Snail mRNA and protein decreased. Data are presented as mean ± SEM. ^*∗*^*p* < 0.05, ^*∗∗*^*p* < 0.01.

**Figure 5:** Schematic diagram of SHH signal pathway on renal fibrosis process.

## Data Availability

The datasets generated and/or analyzed during this study are available from the corresponding author upon reasonable request.

## Abbreviations

CKD: Chronic kidney disease
RIF: Renal interstitial fibrosis
UUO: Unilateral urethral obstruction
TGF-*β*1: Transforming growth factor *β*1
*α*-SMA: *α*-Smooth muscle actin
EMT: Epithelial-to-mesenchymal transition
ECM: Extracellular matrix
ESRD: End-stage kidney disease
SHH: Sonic hedgehog
NRK-49F: Normal rat kidney interstitial fibroblasts
Gli1: Glioma-related cancer gene homologous proteins 1
Snail: Transcriptional factor Snail.
